# Predictive Value of Red Blood Cell Distribution Width in Poststroke Depression

**DOI:** 10.1155/2021/8361504

**Published:** 2021-07-19

**Authors:** Ming Dai, Qiyao Wei, Yuxin Zhang, Chuanqin Fang, Ping Qu, Lei Cao

**Affiliations:** The Second Affiliated Hospital of Anhui Medical University, Hefei 230000, China

## Abstract

**Purpose:**

Red blood cell distribution width (RDW) is increased in a variety of inflammatory-related diseases. However, there is no report of its clinical significance in poststroke depression (PSD). This study explores the clinical significance of RDW in PSD patients.

**Methods:**

A total of 185 patients with first-ever acute ischaemic stroke (AIS) in the Second Hospital of Anhui Medical University were chosen as subjects. A retrospective observational study was conducted from February 2019 to February 2020. PSD patients were diagnosed at 6 months after stroke based on the Diagnostic and Statistical Manual of Mental Disorders-IV criteria. Clinical and laboratory data were obtained from all patients. Coefficient of Variation (RDW-CV) and standard deviation (RDW-SD) were used to statistically report the performance of red blood cell distribution width.

**Results:**

At the 6-month follow-up, 46 patients were diagnosed with PSD. Compared with non-PSD patients, PSD patients exhibited an increase in RDW-CV and RDW-SD, which positively correlated with serum interleukin 6 (IL-6) concentrations. In PSD patients, only RDW-SD demonstrated a consistent positive association with the Hamilton Rating Scale for Depression (HAM-D) scores at 6 months after admission. RDW-CV, RDW-SD, and IL-6 were recognized as independent predictors of PSD. The area under the receiver operating characteristic (ROC) curve (AUC) of RDW-SD was 0.796 (95% CI: 0.731-0.852) for the prediction of PSD, which was superior to that of RDW-CV. The specificity for predicting PSD was 60.43%, and the sensitivity was 91.30% if RDW-SD was higher than 43.80 fL.

**Conclusions:**

RDW-SD is a simple, inexpensive, rapid, and easily accessible parameter that can be used to predict PSD in patients with stroke.

## 1. Introduction

Stroke, a major health problem in both globally developed and developing countries, took 6.24 million lives worldwide in 2005 [1]. Poststroke depression (PSD), characterized by a depressed mood, loss of interest, fatigue, and sleep disturbance, is among the most frequent neuropsychiatric consequences of stroke and affects up to one-third of stroke patients [2]. As a secondary depression, the occurrence of PSD is related to unfavourable outcomes in terms of delayed neurological recovery and a decline in daily living abilities [3]. Additionally, PSD has high mortality and disability rates, thus creating a heavy burden on society [4]. Although the importance of PSD has been recognized for decades and there are several screening tools for PSD [5], many PSD patients are often neglected because no effective biomarker has been established for PSD. In clinical practice, the identification of potentially effective biomarkers for PSD through simple blood tests is the most attractive strategy due to its ability to reduce the time to diagnosis because of high patient acceptability.

Interleukin 6 (IL-6) is produced quickly and transiently during tissue infection and injury and promotes host defense by stimulating acute phase response, hematopoiesis, and immune response [6]. Studies have shown that the expression level of IL-6 in PSD patients is significantly higher than that in non-PSD patients [7], which is extremely important for the treatment and prevention of PSD. A complete blood count (CBC) is one of the most common tests during hospitalization and can easily be obtained by clinicians. As part of the CBC, red blood cell distribution width (RDW) indicates the size variability of red blood cells. Traditionally, anaemia, including iron deficiency anaemia and vitamin B12 deficiency anaemia, is differentially diagnosed with the wide use of RDW [8]. Recent studies have shown that RDW is related to inflammatory conditions in various diseases, such as sepsis, primary Sjögren's syndrome, rheumatoid arthritis, and pulmonary embolism [9–12]. RDW, as a clinical inflammatory marker, has been extensively applied to evaluate the severity and prognosis of manifold diseases because it is noninvasive, rapid, and economic. Notably, recent data from India show the positive association between RDW and the severity of acute ischaemic stroke (AIS) and the potential for RDW to be a useful predictive biomarker for AIS severity [13]. Nevertheless, no clear evidence has yet shown whether RDW can be used to predict the occurrence of PSD among patients with stroke. The main aim of our study is to examine how RDW and PSD are associated at 6 months and then further determine RDW's predictive value for PSD patients.

## 2. Materials and Methods

### 2.1. Patients

A total of 185 patients with first-ever AIS at the Second Hospital of Anhui Medical University between February 2019 and February 2020 were followed for >1 year. AIS patients were diagnosed through clinical and radiological examinations within 24 h after admission in line with the criteria laid down by the World Health Organization. The exclusion criteria for patients were as follows: (i) patients with hypothalamic infarction; (ii) patients who could not complete the neuropsychological test for various reasons; (iii) patients with accompanying brain trauma, cerebral haemorrhage, Parkinson's disease, brain tumour or severe heart, liver, kidney, lung, haematopoietic system, and mental diseases; (iv) patients who died during follow-up; (v) patients with severe depression; and (vi) patients with severe infections and acute inflammatory diseases. The diagnosis of PSD conformed to the Diagnostic and Statistical Manual IV (DSM-IV) criteria for depression. The severity of depressive symptoms was evaluated following the Hamilton Rating Scale for Depression (HAM-D). The study protocol, based on the principles of the Helsinki Declaration, was reviewed by and obtained approval from the Ethics Committee of the Second Hospital of Anhui Medical University.

### 2.2. Records and Assays

Demographic and laboratory data on admission were prospectively collected. A commercially available enzyme-linked immunosorbent assay (ELISA) (human IL-6 ELISA; Colorfulgen) was employed to assay the serum levels of IL-6 in AIS patients. During the assay, standard curves were established for IL-6, and the concentration of IL-6 was calculated according to the standard curve.

### 2.3. Statistical Analysis

SPSS version 16.0 (SPSS, Chicago, IL, USA) or MedCalc statistical software 10.4 (MedCalc, Mariakerke, Belgium) was adopted to perform statistical analysis. Data were compared with the chi-square test or an independent-samples *t*-test as appropriate. A Spearman rank correlation analysis was employed to examine the relationship between RDW and the clinical characteristics of PSD. Factors independently related to PSD were determined by adopting multivariable logistic regression analysis. The efficacy of RDW in predicting PSD was evaluated by conducting receiver operating characteristic (ROC) curve analysis at the 6-month follow-up. *P* < 0.05 indicated statistical significance.

## 3. Results

### 3.1. Patients' Clinical Characteristics

In total, 185 patients with stroke were enrolled in this study. At the 6-month follow-up, 46 (24.86%) patients were diagnosed with PSD. The demographic and clinical characteristics of non-PSD patients and PSD patients are shown in Table 1. An increase in RDW-CV (Figure 1(a)) and RDW-SD (Figure 1(b)) in PSD patients was observed (both *P* < 0.01).

### 3.2. Correlations between RDW-CV, RDW-SD, and the Clinical Characteristics of PSD

In PSD patients, RDW-CV (Figure 2(a)) and RDW-SD (Figure 2(b)) were positively correlated with the serum IL-6 concentrations, with a correlation coefficient of 0.612 for RDW-CV (*P* < 0.001) and 0.458 for RDW-SD (*P* = 0.001). However, only RDW-SD (*r* = 0.304, *P* = 0.040) but not RDW-CV (*r* = 0.116, *P* = 0.443) was positively correlated with HAM-D scores at 6 months after admission, as shown by the correlation analysis between RDW-CV (Figure 3(a)), RDW-SD (Figure 3(b)), and PSD.

### 3.3. Independent Factors Associated with PSD

Univariate and multivariate analyses were used to determine the factors related to PSD. RDW-SD (*P* < 0.001), RDW-CV (*P* = 0.006), IL-6 (*P* < 0.001), and WBC (*P* = 0.007) were associated with PSD, as revealed by univariate logistic regression analysis of the variables. In multivariate logistic regression analysis, only RDW-SD (*P* < 0.001), RDW-CV (*P* = 0.023), and IL-6 (*P* = 0.003) were revealed as independent factors (Table 2).

### 3.4. Predictive Value of RDW-CV and RDW-SD in PSD

An ROC curve was drawn to evaluate the predictive value of RDW-CV and RDW-SD in PSD (Figure 4). The AUC was calculated as 0.634 (95% CI: 0.560-0.703) for RDW-CV and 0.796 (95% CI: 0.731-0.852) for RDW-SD, and the difference in the AUC was statistically significant (*Z* = 4.213, *P* < 0.001). RDW-CV's optimal cut-off value for PSD was 12.6%, with 86.96% sensitivity and 36.69% specificity. RDW-SD's optimal cut-off value for PSD was 43.80 fL, with 91.30% sensitivity and 60.43% specificity.

## 4. Discussion

PSD negatively affects the clinical outcome and prognosis of stroke patients. Its diagnosis is very complicated and is currently only based on clinical parameters. Recent reports have shown that middle-aged PSD patients and stroke survivors without depression have different urine metabolism characteristics [14]. Urine metabolomics can be used to identify potential metabolite markers in patients with poststroke depression in middle-aged patients. PSD patients show a reduction in the gray matter volume (GMV) of the left middle frontal gyrus (MFG), which can provide specific clinical interventions for the treatment of depressive symptoms in poststroke patients.

It is of great significance to predict and identify stroke-stricken patients at high risk for conversion to PSD early, which is the goal of early intervention strategies. However, how to effectively predict PSD remains a challenge. Recently, our efforts have been made to identify biomarkers related to the occurrence of PSD through simple blood tests.

The relationship between inflammation and stroke has been investigated for many years [15–17]. Systemic inflammation is thought to be a risk factor for poststroke complications. Generally, elevated levels of circulating proinflammatory cytokines, including tumour necrosis factor-alpha (TNF-*α*), IL-6, and interleukin 1*β* (IL-1*β*), are related to a poor prognosis in stroke sufferers [18]. Although the pathogenesis of PSD is still unknown, the vital role of inflammation in the onset of PSD has been well established. For example, one study found evidence of a close correlation between the serum level of IL-18 at day 7 poststroke and depression scores at 2 weeks after the initial onset of AIS [19]; another study reported that IL-1*β* and TNF-*α*, as well as their polymorphisms, were involved in the pathogenic process of PSD [20]. Recently, the platelet-to-lymphocyte ratio (PLR) and neutrophil-to-lymphocyte ratio (NLR), as biomarkers conveying information about inflammatory conditions, were proven to be effective predictors of 6-month PSD [21]. The above findings suggest that the inflammatory index could be a significant predictor of the occurrence of PSD.

Similar to the NLR and PLR, RDW is another part of the CBC that could also serve as a biomarker for inflammation-associated processes. It is often expressed as RDW-CV and RDW-SD; the former is the quotient of the standard deviation of the red blood cell volume, whereas the latter is the width of the erythrocyte volume distribution curve at a level 20% above baseline. Recently, several studies have reported the clinical value of RDW in stroke patients. Hong et al. reported an association between RDW-SD and serum NSE levels, which can be considered a risk factor for neuronal damage in AIS patients [22]. The role of RDW-CV as an independent prognostic factor in acute cerebral infarction was revealed by Kim and colleagues [23].

Consistent with these research findings, compared with non-PSD patients, RDW-CV and RDW-SD were significantly higher and positively correlated with serum IL-6 concentrations in PSD patients. Since IL-6 is an inflammatory mediator closely associated with PSD [24], we speculated that elevated RDW-CV and RDW-SD might be observed in patients with stroke who are at high risk for the occurrence of PSD. In PSD patients, RDW-SD was positively correlated with HAM-D scores at 6 months after admission; however, there were no statistically significant correlations between RDW-CV and HAM-D scores at 6 months after admission, implying that RDW-SD may be better suited for predicting PSD in patients with stroke. Subsequently, our study revealed RDW-SD and RDW-CV as independent predictors of PSD. With regard to predicting PSD, the AUCs of RDW-SD and RDW-CV were 0.796 and 0.634, indicating that RDW-SD possesses better predictive value than RDW-CV.

While interpreting the results of this study, several limitations should be considered. This was a single-centre retrospective study with small sample size, suggesting a need for a large-scale multicentre study on stroke patients to support our findings. Due to the short follow-up time, some important factors related to depressive events were not included in the collection, such as the use of antidepressants, psychotherapy, and social support, and these factors may affect the diagnosis of PSD. Nevertheless, our results suggest the potential of RDW-SD to be a marker for the prediction of PSD after acute ischaemic stroke.

Our study confirmed that compared with non-PSD patients, PSD patients exhibited an increase in RDW-CV and RDW-SD, which positively correlated with serum IL-6 concentrations. RDW-SD was positively correlated with HAM-D score, which might be more suitable for predicting poststroke depression in stroke patients. In future clinical work, for patients with AIS, we should focus on the assessment of early depression and pay attention to early psychological intervention and prevention. Early detection and early treatment of PSD will have a good impact on the prognosis of patients.

## Figures and Tables

**Figure 1:** RDW-CV and RDW-SD in non-PSD patients and PSD patients.

**Figure 2:** Correlations between RDW-CV, RDW-SD, and serum IL-6 concentrations in PSD patients.

**Figure 3:** Correlations between RDW-CV, RDW-SD, and HAM-D scores at 6 months after admission in PSD patients.

**Figure 4:** ROC curve for RDW-CV and RDW-SD in PSD patients. The AUC was 0.634 and 0.796, respectively. ROC: receiver operating characteristic; AUC: area under ROC curve.

**Table 1:** Clinical characteristics of patients in this study.

	Non-PSD	PSD	*P* value
Age (years)	62.95 ± 11.34	65.74 ± 10.17	0.140
Gender (female/male)	42/97	12/34	0.709
Education (years)	6.27 ± 4.70	6.17 ± 5.48	0.905
Hypertension (yes/no)	106/33	36/10	0.843
Hyperlipidemia(yes/no)	71/68	25/21	0.736
Diabetes (yes/no)	43/96	15/31	0.856
Coronary heart disease (yes/no)	11/128	7/39	0.158
Atrial fibrillation (yes/no)	6/133	5/41	0.145
Alcohol (yes/no)	37/102	11/35	0.847
WBC (×10^9^/L)	6.66 ± 1.42	7.30 ± 1.11	0.006
IL-6 (ng/L)	35.37 ± 16.38	51.96 ± 27.71	<0.001

**Table 2:** Univariate and multivariate analysis between non-PSD patients and PSD patients.

	Univariate	Multivariate		
	*P* value	Odds ratio	95% CI	*P* value
RDW-CV	0.006	0.434	0.211-0.889	0.023
RDW-SD	<0.001	1.466	1.233-1.743	<0.001
WBC	0.007	1.333	0.997-1.782	0.052
IL-6	<0.001	1.033	1.011-1.055	0.003

## Data Availability

The datasets used and/or analyzed during the current study are available from the corresponding author on reasonable request.

## References

[1] Wafa H. A., Wolfe C. D. A., Rudd A., Wang Y. (2018). Long-term trends in incidence and risk factors for ischaemic stroke subtypes: prospective population study of the South London stroke register. *PLoS Medicine*.

[2] Chen Y. C., Chou W. H., Tsou H. H. (2019). A post-hoc study of D-amino acid oxidase in blood as an Indicator of post-stroke dementia. *Frontiers in Neurology*.

[3] Zhang X., Bi X. (2020). Post-stroke cognitive impairment: a review focusing on molecular biomarkers. *Journal of Molecular Neuroscience*.

[4] Robinson R. G., Jorge R. E. (2016). Post-stroke depression: a review. *The American Journal of Psychiatry*.

[5] Pietra Pedroso V. S. (2016). Biomarkers in Post-stroke Depression. *Current Neurovascular Research*.

[6] Kishimoto T. (2005). Interleukin-6: from basic science to medicine--40 years in immunology. *Annual Review of Immunology*.

[7] Levada O. A., Troyan A. S. (2018). Poststroke depression biomarkers: a narrative review. *Frontiers in Neurology*.

[8] Takeuchi H., Abe M., Takumi Y. (2019). Elevated red cell distribution width to platelet count ratio predicts poor prognosis in patients with breast cancer. *Scientific Reports*.

[9] Ellahony D. M., El-Mekkawy M. S., Farag M. M. (2020). A study of red cell distribution width in neonatal sepsis. *Pediatric Emergency Care*.

[10] Hu Z. D., Sun Y., Guo J. (2014). Red blood cell distribution width and neutrophil/lymphocyte ratio are positively correlated with disease activity in primary Sjogren's syndrome. *Clinical Biochemistry*.

[11] Remalante P. P. M., Salido E. O., Penserga E. G., Gauiran D. T. V. (2020). Red cell distribution width and neutrophil-lymphocyte ratio in rheumatoid arthritis. *Rheumatology International*.

[12] Hammons L., Filopei J., Steiger D., Bondarsky E. (2019). A narrative review of red blood cell distribution width as a marker for pulmonary embolism. *Journal of Thrombosis and Thrombolysis*.

[13] Mohindra R., Mishra U., Mathew R., Negi N. S. (2020). Red cell distribution width (RDW) index as a predictor of severity of acute ischemic stroke: a correlation study. *Advanced Journal of Emergency Medicine*.

[14] Wu J., Wu M., Wu Q. (2020). Identification of potential metabolite markers for colon cancer and rectal cancer using serum metabolomics. *Journal of Clinical Laboratory Analysis*.

[15] Anrather J., Iadecola C. (2016). Inflammation and stroke: an overview. *Neurotherapeutics*.

[16] Jayaraj R. L., Azimullah S., Beiram R., Jalal F. Y., Rosenberg G. A. (2019). Neuroinflammation: friend and foe for ischemic stroke. *Journal of Neuroinflammation*.

[17] Khoshnam S. E., Winlow W., Farzaneh M., Farbood Y., Moghaddam H. F. (2017). Pathogenic mechanisms following ischemic stroke. *Neurological Sciences*.

[18] Li Q., Cao Y., Dang C. (2020). Inhibition of double-strand DNA-sensing cGAS ameliorates brain injury after ischemic stroke. *EMBO Molecular Medicine*.

[19] Yang L., Zhang Z., Sun D., Xu Z., Zhang X., Li L. (2010). The serum interleukin-18 is a potential marker for development of post-stroke depression. *Neurological Research*.

[20] Kim J. M., Kang H. J., Kim J. W. (2017). Associations of tumor necrosis factor-*α* and interleukin-1*β* levels and polymorphisms with post-stroke depression. *The American Journal of Geriatric Psychiatry*.

[21] Hu J., Zhou W., Zhou Z., Han J., Dong W. (2020). Elevated neutrophil-to-lymphocyte and platelet-to-lymphocyte ratios predict post-stroke depression with acute ischemic stroke. *Experimental and Therapeutic Medicine*.

[22] Hong L., Fang K., Ling Y. (2020). Red blood cell distribution width is associated with collateral flow and final infarct volume in acute stroke with large artery atherosclerosis. *Seminars in Thrombosis and Hemostasis*.

[23] Kim J., Kim Y., Song T. J. (2012). Red blood cell distribution width is associated with poor clinical outcome in acute cerebral infarction. *Thrombosis and Haemostasis*.

[24] Zhang X. F., Zou W., Yang Y. (2016). Effects of IL-6 and cortisol fluctuations in post-stroke depression. *Journal of Huazhong University of Science and Technology. Medical Sciences*.

